# Clinical Efficacy and Safety of Tenofovir in the Treatment of Patients with Chronic Hepatitis B

**DOI:** 10.1155/2022/1673453

**Published:** 2022-06-21

**Authors:** Feng He, Zhongjiang Xia, Hui Wang, Jinjun Zhu, Laiwen Hu

**Affiliations:** Department of Infectious Diseases, Anqing First People's Hospital Affiliated to Anhui Medical University, Anqing City, Anhui Province 246000, China

## Abstract

The negative rate of serum HBV DNA, HBeAg, and ALT in the tenofovir group was significantly higher than that in the entecavir group (86.67%, 3.33%, and 80.00%) (all *P* < 0.05). In the tenofovir group, 2cases were considered. *Objective*. The aim of this study is to analyze the clinical effect and safety of tenofovir in the treatment of chronic hepatitis B (CHB) patients. *Methods*. A total of 60 patients with CHB who were admitted and treated in Anqing First People's Hospital Affiliated to Anhui Medical University from January 2019 to July 2020 were randomly assigned at a ratio of 1 : 1 into the tenofovir group (treated with tenofovir) and the entecavir group (treated with entecavir) via the random number table method. The clinical therapeutic effect and safety of the two groups were compared. *Results*. The serum hepatitis B virus (HBV) DNA levels in the two groups decreased after treatment, but there was no significant difference. Ths (2.50%) had nausea, 1 (1.25%) had headache, and 0 had an elevated creatine kinase. In the tenofovir group,1(3.33%) had nausea, 0 had headache, and 0 had an elevated creatine kinase. In the entecavir group, there were 3 (10.00%) cases of nausea, 2 (6.67%) cases of headache, and 1 (3.33%) case of elevated creatine kinase. The overall incidence of adverse reactions in the tenofovir group (3.33%) was significantly lower than that in the entecavir group (20.00%) (all *P* < 0.05). *Conclusion*. Tenofovir is more effective than entecavir in the treatment of patients with CHB due to low incidence of adverse events and a good safety profile.

## 1. Introduction

Chronic hepatitis B (CHB) [1] refers to a chronic liver disease caused by persistent hepatitis B virus (HBV) infection. There were no abnormalities in serum ALT and AST during more than 3 consecutive follow-up visits and a liver histology was expected [2]. Usually, it can be transmitted through blood, mother-to-child transmission, and sexual contact. The clinical manifestations are fatigue, fear of eating, nausea, abdominal distension, pain in the liver area, etc. In severe cases, it may be accompanied by chronic liver disease, spider nevus, abnormal liver function, or persistent abnormality. According to the World Health Organization (WHO), there are about 257 million people with chronic HBV infection globally and about 887,000 people die of HBV infection every year [3]. In 2014, the survey results of the Chinese Center for Disease Control and Prevention (CDC) showed that there were about 70 million cases of chronic HBV infection in the general population in China and 20–30 million of them were CHB patients [4]. HBV replication is closely related to disease progression. Hepatitis B vaccination is currently the most effective prevention method. Due to the low HBsAg clearance rate in CHB patients, no specific drug has been developed to eliminate the virus. Antiviral, liver protection, antifibrosis, and immunomodulatory therapies are the primary treatment methods, which can effectively inhibit the virus replication for a long time, thereby delaying the occurrence of liver cirrhosis and hepatocellular carcinoma. Therefore, the antiviral drugs such as nucleoside (acid) analogs (NA) and *α*-interferon are used. Among them, entecavir (ETV) and tenofovir (TDF) [5] in NA have a strong inhibitory effect on HBV replication and a high resistance gene barrier, which can inhibit the specific binding of HBV polymerase by specifically binding to HBV. It is recommended as a first-line drug [6].

Among all drugs, tenofovir is a new type of nucleotide reverse transcriptase inhibitor, which inhibits reverse transcriptase similarly to nucleoside reverse transcriptase inhibitors. To a certain extent, it can reduce transaminase, protect the liver, and has a good effect on the treatment of hepatitis B. Since the CYP450 enzyme system does not metabolize the drug, there is a possibility of interaction with other medications caused by this enzyme. The low toxicity of this drug enables it to be used in combination with other reverse transcriptase inhibitors in the treatment of hepatitis B [7, 8]. In this study, antiviral drugs combined with Chinese patent medicine Yiganling Soft Capsules were used. Its main ingredient is silymarin, which can improve liver function and protect liver cell membrane. It can be used for acute and chronic hepatitis and persistent hepatitis. It is mainly used to treat a variety of symptoms caused by liver and kidney yin deficiency, unresolved dampness and toxin, and liver discomfort; as in jaundice, anorexia, abdominal distension and bitter taste, fatigue, liver pain, etc. Liver drugs can also be used for the treatment of chronic hepatitis with elevated transaminases. 

## 2. Materials and Methods

### 2.1. Baseline Information

A total of 60 patients with CHB admitted and treated in Anqing First People's Hospital Affiliated to Anhui Medical University from January 2019 to July 2020 were randomly assigned at a ratio of 1 : 1 into the tenofovir group (treated with tenofovir) and the entecavir group (treated with entecavir). In the tenofovir group, the patients were aged 25–65years. In the entecavir group, the patients were aged 24–69years. This study has been reviewed and approved by the Medical Ethics Committee of the Anqing First People's Hospital Affiliated to Anhui Medical University (approval no. AQYY-YXLL-18-19).

### 2.2. Inclusion and Exclusion Criteria

#### 2.2.1. Inclusion Criteria

Inclusion criteria were defined as follows: ① all patients diagnosed with CHB according to the diagnostic criteria of “Guidelines for the Prevention and Treatment of Chronic Hepatitis B (2019 Edition)” [9]; ② normal coagulation; and ③ patients and their families who were aware of the study and voluntarily signed the consent form.

#### 2.2.2. Exclusion Criteria

Exclusion criteria were defined as follows: ① allergic history to research-related drugs, ② combined with mental illness or cognitive dysfunction, and ③ hepatitis caused by other viral infections.

### 2.3. Methods

The entecavir group was given entecavir for treatment, and the patients were orally administered entecavir (Anhui Baker Biopharmaceutical Co. Ltd., H20140037) 0.5 mg/time, once a day, for 36weeks.

The patients in the tenofovir group were treated with tenofovir and oral tenofovir capsules (Chengdu Better Pharmaceutical Co. Ltd., H20163436) 300 mg/time, once a day, for 36 weeks.

At the same time, patients in both groups were given the Chinese patent medicine Yi Liver Spirit Soft Capsules as an adjunctive treatment. Yilanling Soft Capsules (Wuhu Green Leaf Pharmaceutical Company, Z20050476) are to be taken orally, 2 capsules once, three times a day. It is best not to eat cold food or spicy and greasy food during the medication period to avoid irritation of the digestive system or to prevent the absorption of the medicine.

### 2.4. Evaluation Criteria

  â‘Serum HBV DNA level: The Gentier 96 fluorescence quantitative PCR instrument (Xi'an Tianlong Technology Co. Ltd.) was used to detect the serum HBV DNA level.
  â‘¡ Antiviral efficacy : Â The antiviral efficacy of the two groups was evaluated regarding the “Guidelines for the Prevention and Treatment of Chronic Hepatitis B 2015 Edition” [10], and the HBV-DNA negative rate, Hepatitis B e antigen ï1/4ˆHBeAgï1/4‰seroconversion rate, and alanine aminotransferaseï1/4ˆALTï1/4‰ normalization were monitored and compared in the two groups
  â‘¢ Occurrence of adverse reactions: The negative reactions of the two groups of patients during the medication process, such as nausea and headache, were observed and recorded

### 2.5. Statistical Analysis

GraphPad Prism 8 was used to plot graphics, and relevant personnel was used SPSS 22.0 software to process data; count data (*n* (%)) and measurement data (*x* ± *s*) were analyzed using chi-square and *t*-tests, respectively. *P* < 0.05 was considered statistically significant.

### 2.6. General Data Comparison

There was no significant difference in general data between the two groups of patients and they were comparable (see Table 1).

### 2.7. Serum HBV DNA Level

The HBV DNA level of the tenofovir group (0.94 ± 0.28) IU/ml and the entecavir group (1.11 ± 0.44) IU/ml was significantly lower after the treatment. There was no significant difference between the two groups before and after treatment (Figure 1).

### 2.8. Antiviral Efficacy

The negative rate of serum HBV DNA, HBeAg, and ALT in the tenofovir group was significantly higher than that in the entecavir group (6.67%, 3.33%, and 80.00%) (100.00%, 20.00%, and 96.67%) (all *P* < 0.05). See Table 2.

### 2.9. The Occurrence of Adverse Reactions

In the tenofovir group, 1 case (3.33%) had nausea, 0 had headache, and 0 had an elevated creatine kinase; in the entecavir group, there were 3 (10.00%) cases of nausea, 2 (6.67%) cases of headache, and 1 (3.33%) case of elevated creatine kinase. The overall incidence of adverse reactions in the tenofovir group (3.33%) was significantly lower than that in the entecavir group (20.00%) (all *P* < 0.05) (see Table 3).

## 3. Discussion

CHB is caused by infection with HBV [11], a hepatotropic double-stranded linear DNA virus. After being infected with HBV, the patient's liver tissue will be damaged, resulting in inflammatory liver lesions, liver cell swelling, degeneration, and necrosis. HBV infection and replication can lead to excessive deposition of collagen in the necrotic area of the liver, which further develops into liver fibrosis and may eventually progress to liver cirrhosis and liver cancer, thereby aggravating the disease. It is clinically determined that the incubation period of CHB (before the hepatitis virus invades the first clinical symptoms) is about 6 w–6 m, generally 3 m, and the incubation period varies with the type, quantity, virulence, and immune status of the human body [10, 12]. Different outcomes and clinical types may occur after infection with the HBV, host, and environment. At the same time, hepatitis B patients and HBV carriers are the primary sources of infection. According to the epidemiological survey results, about 80% of hepatitis patients in China have viral hepatitis. CHB accounts for about 58% of viral hepatitis and 15%–40% of patients with CHB can develop further. Complications of CHB may occur in fatty liver, liver cirrhosis, hepatic diabetes, post-hepatitis hyperbilirubinemia, etc.

Currently, the clinical treatment principle for CHB includes 30% drug treatment and 70% conditioning [13]. The liver detoxifies many drugs. Excessive use of drugs will increase the burden on the liver, causing relevant diseases. Antiviral drugs are mainly divided into two categories: interferon and nucleotide drugs. Interferon is a glycoprotein that does not directly kill or inhibit the virus but strengthens the activity of human natural killer cells—stimulating macrophages to produce cytokines, enhancing human cellular immune function, killing the virus, and inducing the production of antiviral protein in cells and inhibiting virus replication. Although the interferon has a short course of treatment and a relatively high negative rate of HBsAg, its clinical application is limited due to many disadvantages, such as long-term injection, high price, low compliance, and high adverse reactions. Nucleotide drugs include lamivudine, adefovir dipivoxil, telbivudine, entecavir, tenofovir dipivoxil, tenofovir fumarate, etc. Since these drugs are highly resistant, the guidelines recommend that entecavir and tenofovir dipivoxil be selected as the first-line antiviral drugs in the clinic.

However, no specific drug has been developed to eliminate the hepatitis B virus, so the treatment is still mainly based on antiviral drugs. Therefore, it is of great clinical significance to choose an active and effective antiviral drug for the treatment.

Clinical practice favors entecavir because the triphosphate produced by phosphorylation of entecavir plays an essential role in initiating and reversing transcription of HBV replication. It can effectively inhibit HBV replication and achieve antiviral purposes [14, 15]. Previous research suggests that tenofovir can be phosphorylated to produce diphosphate after being rapidly absorbed by patients orally, and the diphosphate can compete with 5′-deoxyadenosine triphosphate binding. This can effectively prevent the elongation of the DNA chain and finally play an antiviral effect. Both HBV DNA and HBeAg are markers of HBV replication, which can directly reflect HBV replication and proliferation, while ALT normalization can reflect the recovery of liver functions in patients [16]. The combination of traditional Chinese medicine can inhibit or reverse liver fibrosis, effectively inhibit the proliferation of hepatic stellate cells in vivo [9, 11, 12], reduce and activate collagen synthesis, and affect the metabolism of connective tissue. The research shows that after the treatment of hepatitis B decoction combined with tenofovir, the HBV-DNA negative conversion rate, liver function index, and liver fibrosis index of patients have improved. The results once again prove the effectiveness of this treatment method [8].

This study showed that the serum HBV DNA levels in both groups significantly decreased after treatment. The negative rate of serum HBV DNA, HBeAg, and ALT normalization in the tenofovir group was significantly higher than that in the entecavir group. We believe that tenofovir and entecavir are both first-line nucleoside analogues through analysis. However, they can inhibit the replication and synthesis of HBV virus DNA. Their clinical products and competitive mechanisms are not the same. Entecavir is phosphorylated to generate a triphosphate, which competes with the natural substrate of polymerase in the DNA chain of the HBV virus; tenofovir, as a new type of nucleotide reverse transcriptase inhibitor, can directly compete with the deoxyribose substrate. DNA chain extension was performed to achieve the purpose of antiviral treatment. The results are consistent with the results suggested by Peng et al. This study also showed a lower overall incidence of adverse reactions in the tenofovir group, suggesting that tenofovir has a prominent safety profile. It is hardly absorbed through the gastrointestinal tract, so it undergoes esterification and salt formation to become tenofovir disoproxil fumarate and CYP450 enzymes do not metabolize it. Tenofovir also has no interaction with other drugs. The treatment of CHB is a long-term process. Since this study has not yet involved the long-term treatment effect, deficiencies still need to be verified in future studies.

## 4. Conclusion

Tenofovir is safe and reliable and can lower the incidence of adverse events. It is proven to be more effective than entecavir. This study is mainly aimed at the therapeutic targets of drugs. The molecular mechanism of tenofovir on CHB patients is unclear and will be studied in the future.

## Figures and Tables

**Figure 1:** Comparison of serum HBV DNA levels between the two groups of patients. After treatment, tenofovir group serum HBV DNA levels (0.94 ± 0.28) IU/ml and entecavir group serum HBV DNA levels (1.11 ± 0.44) IU/ml were significantly decreased compared with those of tenofovir group (7.45 ± 0.53) IU/ml and entecavir group (7.48 ± 0.67) IU/ml (*P* < 0.05) before treatment, no statistically significant difference. ^*∗*^*P* < 0.05.

**Table 1:** Patient profiles ($\bar{x}$ ± *s*).

Groups	*n*	Male	Female	Age	Average age	BMI
Tenofovir group	30	24	6	25–65	41.90 ± 11.40	22.48 ± 0.64
Entecavir group	30	20	10	24–69	42.10 ± 10.52	22.53 ± 0.59
*t*	—	—	—	—	0.445	0.514
*P*	—	—	—	—	0.657	0.608

**Table 2:** Comparison of antiviral efficacy between the two groups of patients (%).

Groups	*n*	HBV-DNA negative rate	HBeAg negative conversion rate	ALT normalization
Tenofovir group	30	30 (100.00)	6 (20.00)	29 (96.67)
Entecavir group	30	26 (86.67)	1 (3.33)	24 (80.00)
*X* ^2^	—	4.286	4.043	4.043
*P*	—	0.038	0.044	0.044

**Table 3:** Comparison of adverse reactions in the two groups of patients (%).

Groups	*n*	Nausea	Headache	Elevated creatine kinase	Total
Tenofovir group	30	1 (3.33)	0 (0.00)	0 (0.00)	1 (3.33)
Entecavir group	30	3 (10.00)	2 (6.67)	1 (3.33)	6 (20.00)
*X* ^2^	—			4.043	
*P*	—			0.044	

## Data Availability

No data were used to support this study.
